# Interrelationship between Dendritic Cell Trafficking and *Francisella tularensis* Dissemination following Airway Infection

**DOI:** 10.1371/journal.ppat.1000211

**Published:** 2008-11-21

**Authors:** Erez Bar-Haim, Orit Gat, Gal Markel, Hila Cohen, Avigdor Shafferman, Baruch Velan

**Affiliations:** Department of Biochemistry and Molecular Genetics, Israel Institute for Biological Research, Ness-Ziona, Israel; Stanford University School of Medicine, United States of America

## Abstract

*Francisella tularensis*, the etiological agent of the inhalation tularemia, multiplies in a variety of cultured mammalian cells. Nevertheless, evidence for its in vivo intracellular residence is less conclusive. Dendritic cells (DC) that are adapted for engulfing bacteria and migration towards lymphatic organs could serve as potential targets for bacterial residence and trafficking. Here, we focus on the in vivo interactions of *F. tularensis* with DC following airway infection of mice. Lethal airway infection of mice with the live vaccine strain (LVS) results in trafficking of a CD11b^high^/CD11c^med^/autofluorescence^low^ DC subset from the respiratory tract to the draining mediastinal lymph node (MdLN). Simultaneously, a rapid, massive bacterial colonization of the MdLN occurs, characterized by large bacterial foci formation. Analysis of bacteria in the MdLN revealed a major population of extracellular bacteria, which co-exists with a substantial fraction of intracellular bacteria. The intracellular bacteria are viable and reside in cells sorted for DC marker expression. Moreover, in vivo vital staining experiments indicate that most of these intracellular bacteria (∼75%) reside in cells that have migrated from the airways to the MdLN after infection. The correlation between DC and bacteria accumulation in the MdLN was further demonstrated by manipulating DC migration to the MdLN through two independent pathways. Impairment of DC migration to the MdLN, either by a sphingosine-1-phosphate receptor agonist (FTY720) or by the D prostanoid receptor 1 agonist (BW245C), resulted in reduced bacterial colonization of MdLN. Moreover, BW245C treatment delayed the onset of morbidity and the time to death of the infected mice. Taken together, these results suggest that DC can serve as an inhabitation niche for *F. tularensis* in the early stages of infection, and that DC trafficking plays a role in pathogen dissemination. This underscores the therapeutic potential of DC migration impairing drugs in tularemia treatment.

## Author Summary

The high infectivity of *Francisella tularensis* via inhalation led to its classification as a Category-A bio-threat agent and renewed the interest in this pathogen. Here, we characterize early events in respiratory tularemia, which could be instrumental in designing new therapeutic approaches. We focus on the interaction of *F. tularensis* with dendritic cells, which serve as first-line sentinels for invading bacteria and are expected to be pivotal in initiation of host protective response. In this study, we show that lethal airway infection of mice with *F. tularensis* results in accumulation of both bacteria and dendritic cells in the draining lymph node, and that viable bacteria can be detected in dendritic cells that have been recently imported from the airways. The correlation between trafficking of dendritic cell and bacteria is further substantiated by demonstrating that impairment of dendritic cell migration to the draining lymph node through two independent pathways results in decreased bacterial accumulation in the lymph node. Taken together, our observations suggest that *F. tularensis* actually harnesses dendritic cells to facilitate bacterial dissemination and to enhance host invasion. These findings call for examination of the therapeutic potential of drugs that impair dendritic cell migration as countermeasures for tularemia.

## Introduction

Dendritic cells (DC) are a heterogeneous group of antigen presenting cells (APC), which reside in peripheral tissues, and serve as sentinels for invading microorganisms. Most often, contact of DC with microorganisms results in engulfment of the microorganism, and triggers a series of programmed events (maturation). These include surface expression of MHC class II and of co-stimulatory molecules, induction of cytokine secretion, and degradation of the internalized pathogen, allowing for surface-presentation of its antigens to naïve T cells [1].

The encounter between DC and T cells is facilitated by the induced trafficking of activated DC from the periphery to the vicinal draining lymph nodes. The mechanisms that control DC trafficking appear to be complex. Modulation of the surface display of chemokine receptors (up regulation of CCR7 expression and down regulation of other receptors) plays a key role in this process [2],[3],[4]. In addition, other effectors including prostaglandins [5] and sphingosine-1-phosphate [6] also play a critical role in DC migration.

*F. tularensis*, the etiological agent of tularemia, is a zoonotic pathogen with a broad host range. Disease manifestations depend upon the route of infection and include ulceroglandular infection, respiratory infection and a typhoidal disease [7]. The high infectivity of certain *F. tularensis* strains via inhalation led to their classification as a Category-A threat agent. Two subspecies of *F. tularensis*, *F. tularensis* subsp. *tularensis* (type A) and *F. tularensis* subsp. *holoarctica* (type B) are highly infectious to humans yet only the type A bacterium is life-threatening [7],[8]. Most research on the pathogenesis of *F. tularensis* has been performed on mice using the live vaccine strain (LVS) derived from *F. tularensis* subsp. *holoarctica*. This organism shows attenuated virulence in humans but is lethal to mice following pulmonary infection [9].

*F. tularensis* strains are capable of infecting and multiplying in a variety of cultured cells (reviewed in [10]). The mechanisms used by the pathogen to escape the phagocytic pathway and grow inside cells have been the subject of intense research [11],[12], and specific proteins required for intra-macrophage growth were identified. These include members of the *igl*ABCD operon [13],[14] and the *pdp*A and *pdp*D genes contained within a *Francisella* pathogenicity island (reviewed in [15],[16]). In many cases mutant strains that are impaired in intra-macrophage growth were also identified as attenuated in murine infection models [12],[17].

All this led to the accepted notion that intracellular growth is a key mechanism used by *F. tularensis* to escape host defense. Nevertheless, the direct body of evidence for intracellular growth *in vivo* is rather meager. Intracellular LVS bacteria were identified by immunostaining in lungs of infected mice [18] and PCR analyses suggest that practically all *F. tularensis* LVS organisms of bacteremic mice are cell-associated [19]. Nevertheless, the association between LVS and blood cells was recently contested by showing that the majority of *F. tularensis* recovered from blood of infected mice reside in the plasma [20]. Thus, in spite of the increased efforts in this direction, the various manifestations of the interaction of *F. tularensis* with host cells, and the role of these interactions in tularemia pathogenesis are far from being resolved.

In the present study we have focused on the interactions of *F. tularensis* LVS with DC *in vivo*. We show that airway infection by LVS is followed by bacterial colonization of the mediastinal lymph node (MdLN), which occurs in parallel to recruitment of respiratory tract DC (RTDC) from the airways to this draining lymph node. Moreover, administration of two different DC migration inhibitors impairs bacteria accumulation in the MdLN, and not less importantly, affects the course of disease. Finally, we show that cells with characteristic DC phenotype that have immigrated to the MdLN from the respiratory tract carry viable intracellular *F. tularensis*.

## Results

### Pulsing of BMDC by LVS results in intracellular bacterial propagations as well as induction of cell migration

Several aspects of bacteria/DC interactions can affect the dynamics of dissemination in the infected host. Among the most relevant ones are cell inhabitation by bacteria and the ability to trigger DC trafficking. These two features were examined in an in vitro LVS-infection system, using bone marrow DC (BMDC) as target cells.

In accordance with a previous report [21] LVS was found to replicate in BMDC as efficiently as in the macrophage-like J774A.1 cells (Figure 1A). Pulsing of host cells with bacteria (even at an MOI as high as 200) led to an inefficient cell uptake (∼5×10^4^ bacteria were taken up by 10^6^ cells). Yet, once bacteria are taken-up by J774A.1 cells or BMDC, intracellular propagation appeared to be very efficient, resulting in increase of more than two orders of magnitude within 24 hrs.

**Figure 1:** Interaction of BMDC and LVS in vitro Alter. (A) Propagation of LVS in J774A.1 cells and BMDC: Infection was performed as described in the Materials and Methods section, and gentamicin was added 1 hr post pulsing with bacteria. Cells were harvested 2 or 24 hrs post infection, washed, and lysed with DOC. Lysates were diluted and plated for CFU enumeration. Each bar represents the average CFUs in three infection wells. The entire experiment represents one of three repetitions. For visualization of cell-associated bacteria by fluorescence microscopy, infected J774A.1 or BMDC cells were stained with anti-LVS antibodies 24 hrs post LVS infection. (B) Expression of CCR7 by BMDC: Cells were analyzed for CCR7 expression 24 hours post infection with the live or formaldehyde-killed LVS. Non-pulsed cells and cells pulsed with 1 µg/ml *E. coli* LPS served as negative and positive controls, respectively. Gray lines denote isotype-matched immunoglobulin controls. Fractions of CCR7^positive^ cells are indicated. (C) DC were pulsed as indicated above, and expression of co-stimulatory molecules was examined as described in Materials and Methods. Geomeans of fluorescence intensities are presented as relative values, using the values obtained for each marker by pulsing with 1 µg/ml *E. coli* LPS as 100. Results are presented by bar diagrams as the averages of three independent experiments. (D) Migration of BMDC: Cells were pulsed as indicated above, 24 hrs later cells were examined for migration in Transwell chambers towards CCL19 or control medium. Non-pulsed cells and cells pulsed with LPS served as controls. Results are presented as percent cells migrating from the upper compartments to the lower compartment. Each bar represents the average migration in 3 Transwells. The experiment was repeated 3 times. Data presented in this figure were generated by using BALB/c BMDC. Results were confirmed with DC derived from C57BL6 mice.

Induction of maturation responses by *F. tularensis* in APC was examined previously, revealing complex interactions, involving activating as well as inhibitory effects [21],[22],[23]. Acquisition of migratory properties is one of the aspects of bacteria-triggered DC maturation and could, in principal, be also subjected to inhibitory effects by LVS. As a first step in examining the effect of LVS/DC interactions on cell migration we have examined surface expression of CCR7, a receptor involved in DC trafficking from the periphery to lymph nodes [4],[24]. Flow cytometry analysis of pulsed BMDC revealed a notable increase of CCR7 display (Figure 1B and 1C). As expected, LPS of *E. coli*, which served as positive control, led to an effective CCR7 induction. Killed LVS bacteria were also found to be effective, though to a lesser extent, in inducing surface display of CCR7, attesting to the stimulatory potential of LVS pathogen associated molecular patterns (PAMP). Most importantly, live bacteria were as effective as killed bacteria in promoting CCR7 display, arguing against potential abrogating effects exerted by the live pathogen. This is in contrast to the effect of LVS on other markers of DC activation such as TNF-α secretion, where induction occurs with killed bacteria and is abrogated by live bacteria (not shown). It is also interesting to note that display of certain co-stimulatory surface molecules, such as CD83 and CD40 is affected by the viability of LVS (Figure 1C). However, display of other molecules (e.g., CD86) appears to be efficient following pulsing by live as well as killed bacteria.

As an additional step in evaluating DC migratory properties, we have used an in vitro transmembrane chemotaxis assay. BMDC were exposed to various stimulants for 24 hrs and then allowed to migrate through a nylon mesh towards the CCR7-ligand CCL19 (Figure 1D). As controls, we have used non-treated cells and cells exposed to *E. coli* LPS. Pulsing DC with *E. coli* LPS led to effective induction of migration towards CCL19 (6 folds increase over background). Pulsing with LVS bacteria resulted also in induction of cell migration (about 4.5 folds over background). Migration appears to be, at least partly, CCR7-dependent since migration in presence of CCL19 is higher than in its absence (Figure 1D). Again, no differences were found between the effects of killed and live bacteria, suggesting that LVS does not exert adverse effects on DC movement induction.

Taken together, the in vitro analyses suggest that DC have the potential to serve as replication niches, as well as transport vehicles for LVS. This prompted us to examine these functions in vivo.

### LVS colonization of lymph nodes following respiratory infection of mice

The interrelationship between *F. tularensis* and DC in vivo was examined by using a mouse model for respiratory tularemia. As a first step, we have examined the kinetics of LVS dissemination from the respiratory tract to host organs. Mice were infected by intranasal administration of 10^5^ CFU of LVS, which is equivalent to ∼100 LD_50_ (LD_50_ = ∼1000 CFU, our results as well as those of others [9]) leading to death within 5–6 days.

Intranasal administration of LVS resulted in robust proliferation of the bacterium in the airways (Figure 2A), confirming earlier reports [25],[26]. Bacterial counts in lungs increased by at least three orders of magnitude within 2 days and remained constant as long as mice were alive (Figure 2A). As expected, immediately after infection, bacteria were localized in the broncholaveolar lavage fluid (BALF). In the following days bacterial counts in the lung were divided equally between BALF and lung tissue, and during the late days of infection the relative amount of BALF bacteria was somewhat lower (Figure 2A).

**Figure 2:** Spreading of LVS in intranasally infected mice. Mice were infected intra-nasally with 10^5^ CFU of LVS. (A) Bacteria were counted in BALF, lung tissue after lavage, MdLNs, spleens, and livers in animals sacrificed at the indicated time points after infection. Single cell suspensions derived from the various organs were diluted in PBS and plated for CFU counts. Each bar represents the average counts in 3 individual animals. Experiment was repeated 2 more times, resulting in similar observations. (B) Microscopy evaluation of MdLN colonization was performed on cryo-sections of MdLN, 72 hrs post infection with LVS. Sections were stained with rabbit anti-LVS hyperimmune serum and FITC-conjugated secondary antibody. One representative large infection focus is shown.

Monitoring mediastinal lymph node (MdLN) colonization, 24 hrs pot infection revealed viable bacteria, at levels as high as 10^4^ CFU/MdLN (Figure 2A). This number increased to about 10^6^ CFU/MdLN on the second day and then remained unchanged. The accumulation of bacteria in the spleen and liver lagged behind their accumulation in the MdLN. Levels comparable to those found in MdLN at 24 hrs were reached in these organs 48 hrs post infection (Figure 2A).

Taken together, these results underline the role of the draining lymph nodes in respiratory LVS infection. MdLN colonization begins very early post airway infection. It occurs immediately after colonization in the primary infection site (lung), and precedes the spreading of the pathogen to distant organs such as spleen and liver (Figure 2A). The rate of LVS accumulation in the lymph node is very rapid, close to two orders of magnitude within 24 hours, resembling LVS propagation in tissue cultures at optimized conditions (compare Figure 1A and Figure 2A). It is interesting to note that the maximal number of organ-associated bacteria in MdLN is 10^6^ CFU/organ, compared to 10^7^CFU/organ in spleens and livers, which are about 100 folds larger in size.

To better characterize the robust colonization of the draining lymph nodes by LVS, we searched by light microscopy for bacterial localization in cryo-sections of MdLNs 72 hrs post airway infection. This led to identification of distinct bacteria-containing infection foci in LVS infected MdLNs. Most notable are rare (1–2 per cross section), yet very expanded foci carrying a large number of bacteria (Figure 2B). The average number of LVS per cross section of such a focus was found to be 100–200 (such large clusters could not be revealed 24 hrs post infection). Simple geometrical calculations suggest the presence of more than 10^3^ bacteria per one global focus. This morphological feature implies an in-situ clonal expansion of bacteria that have entered the lymph node at an early stage. Thus, bacterial accumulation in the MdLN is not a mere reflection of bacterial influx from other organs. It should be noted that at the same time point (72 hrs post infection), one could find also much smaller foci (not shown) that could have been formed by bacteria entering the MdLN at a later stage.

Taken together, our observations suggest that colonization of the draining lymph node is a major step in bacterial dissemination, following airway infection with LVS.

### LVS infection triggers recruitment of DC to the mediastinal lymph node

Once the kinetics of bacterial spreading was defined, we have examined the cellular events related to respiratory infection of mice by LVS. We have focused on phagocytic cells of the monocytic lineage, and restricted the study to the early infection sites: the respiratory tract and the MdLN.

In general, the respiratory tract monocytic phagocytes can be defined by surface display of two markers, CD11c and CD11b [4],[27] and can be differentiated into alveolar macrophages and pulmonary DC by virtue of their autofluorescence (AF) level. Macrophages are defined by high AF, whereas pulmonary DC exhibit low AF [28].

Analysis of single cell suspensions derived from the MdLN, two days post intranasal infection revealed the presence of cells that are CD11c^med^/CD11b^high^ (Figure 3A, top), of cells that are CD11c^med^/AF^low^ (Figure 3A, center), as well as of cells that are CD11b^high^/AF^low^ (Figure 3A, bottom). These three populations are represented at comparable levels (∼7%), attesting to the presence of a CD11c^med^/CD11b^high^/AF^low^ cell population in the MdLN. The appearance of such cells in the MdLN is infection-dependent, since background levels of this population are ∼10 times lower in non-infected animals (Figure 3A, left panels), as well as in mock infected mice (PBS instillation, not shown).

**Figure 3:** Definition of cell phenotypes in infected lungs and MdLNs. Single cell suspensions of MdLN (A), washed lung (B), and BALF (C) were prepared from organs collected 48 hrs post infection with 10^5^ CFU of LVS. Cells derived from non-infected animals served as controls. MdLN and BALF cell suspensions were stained for expression of CD11c and CD11b using antibodies conjugated to APC or PE, and analyzed by flow cytometry for surface display of markers as well as autofluorescence at FL1. Data are presented in the form of dot diagrams using parallel gating for identification of infection-triggered recruitments (numbers indicate percentage representations of the gated populations). Isotype-matched antibodies served as controls, and the same gates used in specific stain analysis were evaluated. In this case, gated population frequencies in infected organs were comparable to backgrounds (not shown). All analyses presented were conducted on tissues pooled from 3 individual animals. Three independent experiments exhibited similar cell profiles.

The phenotype of the CD11c^med^/CD11b^high^/AF^low^ cell identified in the MdLN matches accurately the phenotype of an identical population, identified in lung tissue (plotting of CD11b vs. AF is shown in Figure 3B). The appearance of this population in the lung is not dependent on infection.

Analysis of cells derived from the BALF revealed this same population, but also revealed a distinct population of CD11b^med^/AF^high^ cells (Figure 3C) which happens to be also CD11c^high^ (not shown). The phenotype of these CD11c^high^/CD11b^med^/AF^high^ cells and their presence in the BALF prompted us to define them as alveolar macrophages (AMΦ). The CD11c^med^/CD11b^high^/AF^low^ population, on the other hand, was defined as a subset of respiratory tract DC (RTDC), relying on previous characterizations of such populations [4],[28]. The definition of these cells as DC is further supported by surface expression of MHC class II (not shown).

The kinetics of RTDC recruitment to the MdLN following infection with 10^5^ CFU of LVS is marked by a burst in cell influx on day 2 (Figure 4) reaching levels close to 10^5^ RTDC per lymph node. This is followed by a decline at later days. The representation of RTDC cells on the first day post infection with 10^5^ CFU was not higher than background levels measured in non-infected mice (Figure 4). Nevertheless, when infection dose was increased from 10^5^ to 10^7^ CFU, one could clearly detect recruitments of RTDC, as early as 24 hours post infection (not shown).

**Figure 4:** Cell recruitment to MdLN following airway infection with LVS. MdLNs were isolated at various time points after intra-nasal infection of mice. Single cell suspensions were analyzed by flow cytometry as indicated on the legend to Figure 3. Number of AMΦ and RTDC at different time points post infection are presented as bar diagrams.

In order to define the origin of the DC imported to the MdLN, we have labeled the respiratory tract cells by vital staining [29]. The orange cell tracer CMTMR was administered to mice by intranasal instillation, five hours prior to intranasal infection by LVS. MdLN cells were isolated on the next day, and examined for presence of CMTMR and for DC-marker expression. In this protocol we have used an infection dose of 10^7^ CFU, which allowed early monitoring of cell trafficking. Flow cytometry analysis revealed MdLN cells carying CMTMR, which also express CD11c (Figure 5A and 5B). One such cell population which is CMTMR^+^/CD11c^med^ exhibits a ∼4 fold increase following infection, indicating migration of CD11c^med^ cells from the respiratory tract to the draining lymph node (Figure 5A and 5B). This migration is substantiated by another set of experiments indicating that the CD11c^med^ cells accumulating in the infected MdLN display on their surface CCR7 (not shown).

**Figure 5:** Identification of cells immigrating from airways to the MdLN by in vivo viable staining. Airway cells of live mice were stained by instillation of CMTMR. Migration to lymph node was induced by intranasal infection with 10^7^ CFU of LVS, using PBS instillation as control. Single cell suspensions were prepared from a pool of 8 lymph nodes collected 18 hrs post infection. Cells were analyzed by flow cytometry prior to (top panel, A and B) or after sorting by MACS with CD11b-microbeads (lower panel, C–F). Cells were stained with either APC-conjugated anti-CD11c (A,B,D,F) or APC conjugated anti-CD11b (C,E). Surface marker staining was plotted against CMTMR staining. Data are presented as dot diagrams. Gating for CMTMR staining and marker staining was based on diagrams of the appropriate non-stained controls (not shown). Numbers indicate cell percentage of the gated populations or of that defined by quadrants. Similar results were obtained in two other similar experiments.

To further characterize the immigrating cells we have fractionated MdLN cells by magnetic sorting (MACS), using beads coated with anti-CD11b antibodies. Bound and non-bound cell fractions were then analyzed for presence of CMTMR and for surface display of CD11b or CD11c (Figure 5C–5F). Sorting by anti CD11b-coated beads resulted in the expected enrichment for cells expressing CD11b but at the same time in enrichment for cells stained by CMTMR (Figure 5C). Actually 27% of the cells in the CD11b-sorted population were highly positive for both CMTMR and CD11b, as opposed to ∼2% in the non-bound fraction (Compare Figure 5C and 5E). Sorting by CD11b also resulted in a comparable enrichment for cells that were CD11c positive (Figure 5D and 5F), leading to 23% representation of CMTMR^+^/CD11c^+^ cells (Figure 5D). Moreover, closer examination of the sorted cells reveals a correlation between high uptake of the viable dye and intermediate expression of CD11c.

The viable staining experiments provide indication to the trafficking of cells expressing both CD11c and CD11b from the respiratory tract to the draining lymph node in the infected animal. This result together with the observed accumulation of RTDC in the infected MdLNs attests to an LVS-induced trafficking of DC *in vivo*.

### Association of LVS with CD11c/CD11b cells within mediastinal lymph nodes

The in vivo trafficking of both viable LVS (Figure 2) and of DC to the MdLN (Figure 5) as well as the in vitro infection results (Figure 1), led us to search for association between host cells and LVS in the infected lymph node.

As a first step in evaluating the localization of bacteria in the MdLN cells, we have subjected single-cell suspensions, obtained 48 hours post intranasal infection, to a gentamicin protection test. About 10% of the bacteria found in the cell suspensions survived gentamicin treatment (Figure 6A), suggesting that this bacterial population is localized within cells and is therefore not accessible to the antibiotic. The other approach used to identify cell-associated bacteria was based on differential centrifugation and provided similar results. Mild spinning (200 g, 10 min) resulted in a supernatant containing ∼90% of the MdLN bacteria and a cell pellet containing ∼10% of the bacterial content (Figure 6A).

**Figure 6:** Association of LVS with a specific cell population in infected lymph nodes. Mice were infected intra-nasally with 10^5^ CFU of LVS. Forty-eight hours later MdLNs were collected from 10 animals and single cell suspensions were prepared and examined by several assays. (A) Association between viable bacteria and MdLN cells was assayed by examining non-washed (total LN suspension) and washed cells for presence of viable LVS prior or post gentamicin treatment. Bacterial counts are presented as CFU per a single MdLN. (B) Association between LVS and RTDC cells was assayed by subjecting the washed cell fraction (∼10^8^ cells) to sorting by magnetic microbeads coated with either anti-CD11b (B, top panel) or anti-CD11c (B, lower panel). Viable bacteria (no gentamicin treatment) were counted in the input cell suspension, in the bound cell fraction, as well as in cells that did not bind to the microbeads, and presented as CFU/10^6^ cells. The amounts of cells in the input and in the bound fractions were ∼10^8^/10 MdLNs and in the bound fractions only ∼10^6^/10 MdLNs. CD11b and CD11c sorted cells were also examined by fluorescence microscopy for presence of intracellular bacteria. Typical cells carrying bacteria are presented in the insets to (B). (C) The cell/bacteria association in the CD11b-sorted fraction was characterized by determining bacterial count in non-treated cells, in cells treated with gentamicin (genta), in cells treated with gentamicin followed by washing and saponin lysis (genta+sap), as well as in cells where saponin treatment preceded gentamicin treatment (sap+genta). All bacterial counts were performed in triplicates, error bars represent variation of these counts. Data presented in this figure were collected from a single experiment. Two additional CD11b sorting experiments and one additional CD11c sorting experiment were conducted, exhibiting similar enrichment of intracellular bacteria.

To characterize the cells that carry LVS, we have subjected washed MdLN cell suspensions to magnetic cell sorting by beads conjugated to anti-CD11b antibodies (Figure 6B, top panel). Fractionated cells were then analyzed for association with LVS. The amount of viable bacteria, per a given number of anti-CD11b bound cells was found to be 1000 folds higher than that in the unbound fraction (Figure 6B, top). Moreover, the actual amount of bacteria in the unbound fraction is in good agreement with the residual amount of ∼0.5% CD11b^+^ cells found in this fraction (data not shown). Altogether this suggests a specific association between LVS and CD11b^+^ cells in the infected lymph node.

Flow cytometry analysis of the CD11b-MACS sorted cells revealed that, as expected (Figure 3 and Figure 5), bound cells display on their surface CD11c in addition to CD11b. This led us to sort infected MdLN cells by anti-CD11c microbeads as well (Figure 6B, bottom panel). Results of this fractionation were very similar to those obtained by CD11b MACS sorting (compare top and bottom panels of Figure 6B). The amount of viable bacteria, per a given number of anti-CD11c bound cells was found to be ∼500 folds higher than that in the unbound fraction (Figure 6B, bottom). Thus, LVS appears to associate with CD11b^+^ as well as CD11c^+^ cells.

In order to determine if the observed bacteria/cell association reflects intracellular residence of LVS, CD11b sorted cells from infected MdLNs were subjected to gentamicin protection tests (Figure 6C). The number of viable bacteria was not affected by pretreatment with gentamicin, indicating that LVS indeed resides inside CD11b^+^ cells. Moreover, when gentamicin-treated cells were lysed with saponin, the number of measurable viable counts was higher by ∼4 folds, indicating presence of several bacteria within one cell. As expected, lysis of cells prior to antibiotic treatment, relieved cell protection, and rendered all bacteria sensitive to gentamicin.

To substantiate the intracellular localization of bacteria in DC of infected lymph nodes, the CD11b sorted cells, as well as CDb11c sorted cells were stained with antibodies specific to LVS. Microscopic analysis revealed cells carrying LVS (Figure 6B, insets). These cells were not very abundant; nevertheless, in almost all cases more than one bacterium was associated with a single cell.

Taken together, the results presented in Figure 6 reveal that viable LVS bacteria reside within MdLN cells that exhibit an RTDC phenotype.

### Association of LVS with newly immigrating cells within the MdLN

To examine the origin of the CD11b-sorted, LVS-carrying cells, we have resorted to in vivo vital staining. Cells lining the respiratory tract were stained with CMTMR, as described above (Figure 5), animals were sacrificed 2 days later, and single cell suspensions derived from the infected MdLNs were first subjected to flow cytometric analysis (Figure 7A). The bound fraction contained, as expected, a substantial amount of fluorescent cells, about 20% of which exhibited fluorescence levels higher then background autofluorescence. These and were therefore defined as CMTMR stained cells (Figure 7A). Only trace amounts of this population were present in the non-bound fraction.

**Figure 7:** Association of LVS with newly immigrating cells in infected lymph nodes. Airway cells of live mice were stained by instillation of CMTMR. Migration to lymph node was induced by intranasal infection with 10^5^ CFU of LVS. Single cell suspensions were prepared from pools of 8 lymph nodes, collected 48 hrs post infection. Cells were sorted by MACS with CD11b-microbeads. Bound and non bound cells were analyzed by flow cytometry (A) to evaluate the fraction of CMTMR^+^/CD11b^+^ cells. Sorted cells were examined by florescence microscopy for presence of the indicated cell phenotype (B). Large numbers of cells were screened to determine the proportion of the various cell populations (C). In addition, the average number of bacteria per cell in LVS-bearing CMTMR^+^ and CMTMR^−^ cells was determined (C, last column).

Sorted cells were mounted on chamber slides, and were screened by fluorescence microscopy for the presence of the intracellular orange CMTMR staining, as well as presence of cell-associated bacteria. This resulted in identification of CMTMR^+^/LVS^+^ cells, CMTMR^+^/LVS^−^ cells, and CMTMR^−^/LVS^+^ cells (representative cells are shown in Figure 7B). The relative distribution of these cell types (Figure 7C) revealed a strong linkage between CMTMR staining and presence of intracellular bacteria. Screening of 1000 cells which were not bound to CD11b, failed to reveal any CMTMR^+^ cells, and revealed only two CMTMR^−^ LVS-carrying cells. Screening of 2200 CD11b-bound cells revealed 220 cells that carried CMTMR at levels sufficient to allow microscopic detection. Of these CMTMR^+^ cells, as much as 38% were found to carry bacteria. In contrast, only 2.5% of the CD11b-bound cells, which were not stained by CMTMR were found to carry bacteria (Figure 7C).

To further define the intra-cellular residence of LVS, we counted the number of bacteria in the individual cells. The average number of bacteria in the CMTMR^+^ cells was found to be 5.2±3.5, and that in the CMTMR^−^ cells 2.8±1.9. When the total number of bacteria residing in these two cell populations is calculated (440 in CMTMR^+^ cells and 140 in CMTMR^−^ cells), it becomes evident that as much as 75% of the bacteria associated with CD11b-sorted cells reside within newly imported cells.

While the actual number of bacteria per cell in the CMTMR^−^ population does not seem to be very different from that in the CMTMR^+^ population (2.8 vs 5.2), the statistical significance of the difference is very impressive (*P*<10^−5^, Figure 7C). This implies that the events leading to bacterial residence in these two cell populations are different.

Taken together, these results attest to preferential bacterial residence in cells that have recently immigrated from the airways to the MdLN. These results also imply that two cell-infection mechanisms take place during airway infection; one occurs in the airway at the early stages of infection, and the other occurring later on, either in the airways or in the lymph node.

### Treatment with the S1P homologue FTY720 results in impairment of DC migration and of MdLN colonization

The residence of intracellular bacteria in RTDC, and more specifically in newly-immigrated MdLN cells suggests that DC play a role in *F. tularensis* trafficking. To further examine this point, the effect of RTDC migration-impairment on bacterial dissemination was tested using FTY720 (fingolimod), a sphingosine analogue. FTY720 counteracts the functions of the sphingosine-1-phosphate (S1P), and thereby impairs cell migration [30]. FTY720 inhibits lymphocyte egress from lymphoid tissue, and was also found to inhibit migration of lung DC to the MdLN [6].

FTY720 in its carrier solution, or carrier solution alone were administered intranasally to mice, concomitantly to infection. MdLNs were analyzed two days later by flow cytometry. The MdLN of infected, mock-treated, animals carried the distinct CD11b^high^/autofluorescence^low^ cell population (Figure 8A), which defines RTDC recruitment (Figure 3). In mice treated with FTY720, this population was brought down to background levels (Figure 8B and 8C), indicating that FTY720 impairs very effectively the LVS-triggered RTDC migration to the MdLN.

**Figure 8:** The effects of FTY720 on accumulation of RTDC and LVS in the MdLN. Mice infected with 10^5^ LVS were treated with FTY720 diluted in carrier solution, or with carrier solution alone, as described in Materials and Methods. To examine DC trafficking, MdLNs were collected 48 hrs post infection and analyzed for RTDC representation (CD11b^high^/autofluorescence^low^) as described in the legend to Figure 3. An experiment was conducted on MdLN pools, each consisting of 6 organs. MdLNs were derived from infected mice treated with either carrier alone (A) or with FTY720 (B). Non-infected, FTY720-treated mice (C) served as controls. Bacterial colonization of the MdLN (D) was examined 48 hrs post infection in each one of the 6 individual FTY720- treated and 6 mock-treated mice, *P*<0.01. Three independent experiments, each conducted with groups of six mice, exhibited similar correlation between RTDC and LVS recruitment.

The FTY720 treatment resulted also in a substantial reduction in the LVS counts in the MdLN (Figure 8D). Mock-treated mice carried 1.3×10^6^±0.9×10^6^ live LVS in the MdLN. This number was reduced by two orders of magnitude in FTY720 treated mice, reaching values of 1.1×10^4^±0.5×10^4^. Thus, administration of a S1P analogue to the airways of LVS infected mice impairs effectively recruitment of RTDC to the MdLN, as well as colonization of this organ, implying that these two events are linked.

### Impairment of DC trafficking by the prostaglandin analogue BWC245C affects MdLN colonization by LVS and disease progression

To substantiate the observed correlation between DC and LVS trafficking, we examined the effects of an additional inhibitor of DC-migration, which is known to act through a different mechanism. We have chosen BW245C, a D prostanoid receptor 1 (DP1) agonist, known to inhibit in vivo migration of Langerhans cells [31],[32] as well as airway DC [5].

BW245C was administered by two intranasal instillations, one immediately prior to LVS inoculation, and the other 24 hours later. The effect of agonist administration on recruitment of DC and bacteria to the MdLN was examined 48 hours post infection. The BW245C treatment resulted in a marked reduction in the representation of RTDC in the infected lymph node (Figure 9A). While ∼7×10^4^ of the MdLN cells exhibited the RTDC phenotype in LVS infected mice, DC representation in infected mice, treated with BW245C was reduced to ∼2×10^4^. It should be noted that background levels in non-infected mice, either treated or not treated with the agonist, remained ∼0.6×10^4^.

**Figure 9:** The effects of BW245C on the outcome of LVS infection. Mice infected with 10^5^ LVS were treated with BW245 diluted in carrier, or with carrier alone, as described in Materials and Methods. To examine DC trafficking (A), MdLNs were collected 48 hrs post infection and analyzed for RTDC representation (CD11b^high^/autofluorescence^low^). Experiments were conducted on MdLN pools, each consisting of 6 organs, derived from infected or non-infected mice treated with either BW245C or carrier alone. Results are presented by bar diagrams as the averages of three independent experiments. * *P*<0.05. Bacterial colonization of the MdLN (B) was examined 48 hrs post infection in 13 individual BW245C-treated and 13 mock-treated mice. ** *P*<0.05. The effect of BW245 on mortality (C) was examined in groups of 10 mice comparing treated (open squares) and mock-treated mice (closed circles). The experiment presented represents one of three similar experiments. The effect of the drug on morbidity (D) was examined by monitoring weight loss for 5 consecutive days in groups of 10 mice each (8-week-old females). Groups consisted of non-infected BW245-treated mice (closed triangles), infected and treated mice (open squares), and infected mock-treated mice (closed circles). Data are presented as percentage of the weight determined on day zero and calculated separately for each individual mouse. *** *P*-values on days 2–5 range between <0.01 and <0.05.

The effect of BW245C on the infection-dependent DC recruitment was accompanied by a significant impairment of MdLN colonization by LVS (Figure 9B). The average number of viable bacteria in the draining lymph nodes 48 hours post airway infection was 480.000±180.000. This number was reduced to 75.000±21.000 upon treatment with BW245C. It should be noted that treatment had no effect on the number of bacteria or of DC in the lung, excluding possible bacteriostatic/bacteriocidic or cytotoxic effects of the drug in vivo. Taken together, these results provide additional evidence to the linkage between the accumulation of RTDC and of viable bacteria in the draining lymph nodes following infection.

To examine the effect of the DP1 agonist on the course of experimental respiratory tularemia, infected mice were subjected to a short treatment by intranasal instillation of BW245C as described above. Animals were monitored for survival in comparison to infected, sham-treated (instillation of carrier only) animals. Results presented in Figure 9C indicate that the short treatment (day 0 and day 1) resulted in a delay of one day in the time to death of mice. Mean time to death without treatment was 6.4, as compared to 7.5 following treatment. This difference appears to result from a treatment-dependent delay in the onset of the disease manifestations. Monitoring of animal morbidity revealed significant differences (Figure 9D) in the kinetics of weight loss in treated vs. non-treated mice. The first day is marked by a moderate weight loss in all animals, which stems from the instillation procedure itself, as the same loss is also observed in treated non-infected mice. Nevertheless the disease-induced weight loss starts after day 1 in infected non-treated animals and after day 2–3 in treated animal (Figure 9D). Similar experiments, conducted with FTY720 were marred by the intrinsic long-term pleotropic effects of this agonist on lymphocyte mobilization [30]. A single FTY720 instillation into infected animals resulted in a somewhat prolonged mean time to death, but did not alleviate weight loss (not shown).

In summary, treatment with a DP 1 agonist, like treatment with an S1P analogue has a marked effect on DC recruitment to the draining lymph node and on bacterial colonization of the lymph node. This treatment also delays the time point at which disease becomes apparent, and the time of death of the infected animals.

## Discussion

DC play a key role in surveillance for pathogen invasion through skin and mucosal epithelium. DC are highly adapted for sampling, killing and processing microbes, and for trafficking the processed material to regional lymph nodes for antigen presentation.

Impairment of certain DC functions by pathogens has been addressed by numerous studies during the last years (reviewed in [33]), yet much less is known about the specific interplay between DC migration and microbial infection. One can envision two ways by which manipulation of DC migration could enhance microbial invasiveness. DC/pathogen interaction could impair DC migration to the draining lymph node [34],[35], and thereby interfere with the onset of immune responses. Alternatively, hijacking of the DC migration process by intracellular pathogens and its adaptation for dissemination of live microbes [36],[37] could provide an advantageous mechanism for subverting the immune system, and at the same time facilitate the progress of infection.

In the present study we examined the dynamics of DC trafficking in mice infected with *F. tularensis* LVS. It is widely accepted that bacterial PAMP trigger migration of DC through TLR-mediated induction of surface display of the chemokine receptor CCR7. The ability of live LVS to trigger this process is not self-evident. LVS carries on its surface an atypical LPS which is limited in its capacity to interact with cellular TLRs [38],[39],[40], and could therefore be handicapped in triggering signal transudation involved in cell trafficking. Moreover, LVS can actively abrogate activation processes within immune cells, as indicated by the observed effect of live LVS on expression of certain co-stimulatory DC markers (Figure 1C), as well as on expression of pro-inflammatory cytokines (our unpublished results and those of others [22],[23]). In spite of all this, pulsing of BMDC in vitro with LVS resulted in induction of notable, surface expression of functional CCR7 (Figure 1B and 1D).

To examine manifestations of these migratory properties in vivo, a mouse model based on airway infection of mice by LVS was employed, and migration of DC from the infection site to the draining lymph node was analysed. Identification of such DC is complicated by the unique features of respiratory tract APC. Several populations of monocytic phagocytes were identified in the different anatomical compartments of lung [27],[41], and moreover, APC in the pulmonary tract exhibit unusual phenotypes. On one hand, CD11b which is considered to be a typical marker for macrophages, is low in alveolar macrophages yet appears on certain pulmonary DC. On the other hand, CD11c which is routinely used as marker to identify DC in peripheral lymphoid organs is also present on pulmonary macrophages (reviewed in [42],[43],[44] ).

In an attempt to define RTDC populations affected by LVS we have examined lungs of infected mice for expression of CD11c and CD11b and identified two major integrin-expressing populations. One population that is present only in the BALF is characterized by high expression of CD11c, low expression of CD11b and high autofluorescence (Figure 3B) and thus exhibits the characteristics of alveolar macrophages. The other major population can be defined as a RTDC subset (Figure 3A and 3B), as it exhibits low autofluorescence [28],[45], high CD11b expression [4],[46],[47], intermediate level of CD11c [48],[49] and also high surface expression of MHC class II (not shown) [50].

The phenotypic definition of the relevant cell populations (Figure 3), prompted us to search for cell trafficking to the MdLN. This led to the identification (Figure 4) of infection-dependent recruitment of RTDC to the draining lymph node, with no apparent recruitment of AMΦ. Moreover, our experiments suggest that cells have been imported from the infected respiratory tract. The phenotype of the cells matches accurately the phenotype of DC identified in lung tissue and BALF (Figure 3), and cells were shown to carry a vital dye (CMTMR), instilled into the respiratory tract prior to infection (Figure 5).

Taken together our findings indicate that in vivo interactions between *F. tularensis* and DC can induce the signaling process leading to cell migration from the infection site to the draining lymph node. This observation substantiates the prevailing notion that DC but not macrophages are the primary migratory APC following invasion of the airways. We show that such a migration is induced not only by soluble antigens [50] and inert particles and spores [4],[51], but also by viable respiratory pathogens. Moreover, the DC that take part in this process are identified as a specific subset of CD11c^med^/CD11b^high^ RTDC. The CD11b^high^ DC-subset was recently distinguished functionally from the CD11b^low^ subset, and was associated with directing leukocyte trafficking during lung inflammation [37],[46],[52].

Another part of this study was dedicated to bacterial spreading following airway infection with LVS (Figure 2A). We show that infiltration of MdLN by bacteria is a very early event (occurring during the first day of infection), resulting in a massive load of bacteria accumulating in the lymph node, at a very high rate (Figure 2A). These results, which characterize infection by LVS as well as by the Schu4 strain [22] suggest that colonization of draining lymph nodes is an important stage in bacterial spreading. Moreover, microscopic analysis of MdLN from LVS infected mice at the late stages of infection reveal large foci of infection carrying tens of bacteria, suggesting in situ replication of a clonal nature, *i.e.* single bacteria infiltrating the tissue at early stages have replicated in the lymph node to generate a large condensed focus. All this underlines the major role played by tropism for lymphatic organs in *F. tularensis* pathogenesis.

It is tempting to speculate that the invading bacteria are carried into the MdLN by immigrating RTDC. The rate of bacterial spreading from the infected airways actually supports such a model. Bacteria can be detected in MdLNs at substantial amounts, as early as 24 hrs post infection, and this correlates well with short time frames reported for transport of soluble or particulate antigen from the airways to the draining lymph nodes in mice [4],[50],[51],[53]. Nevertheless, comparison of the kinetics of bacterial inhabitation of the MdLN to those of DC recruitment reveals that bacteria are detected in the lymph node at least one day prior to a notable increase in DC numbers (compare results of infection with 10^5^CFU in Figure 2A and Figure 4). One should note, however, that the sensitivity of detecting bacterial import is much higher than that for detecting DC import. One can easily detect the presence of several CFU in the MdLN, whereas detection of newly immigrating DC over a background of ∼1% representation is difficult (Figure 3A and Figure 4). Actually, one cannot preclude the possibility that LVS infection triggered the immigration of ∼10^3^ DC (∼10% of the observed background) on the first day of infection and that these cells are instrumental in spreading the infection. Indeed when intranasal infection dose was increased from 10^5^ to 10^7^ CFU newly immigrating DC were identified 24 hrs post infection (Figure 5), indicating that early recruitment does occur, and suggesting that the extent of recruitment is dependent on the bacterial load in the respiratory tract.

As a first step in defining the correlation between LVS and DC accumulation in the draining lymph node, we have identified intracellular inhabitation of LVS in MdLN cells. LVS-carrying cells could be enriched by magnetic sorting for expression of CD11c as well as CD11b. The similar efficiency of the two sorting processes (Figure 6B and 6C) in retrieving cell-associated bacteria suggests that LVS-containing cells express CD11c as well as CD11b on the same cell. CD11c and CD11b expression, which characterizes monocytic phagocytes is not exclusive to DC, yet presence of such cells in MdLNs following airway infection would argue for their definition as RTDC [4]. The cell-associated bacteria were found to be viable, as indicated by their ability to form colonies and are located within the cells, as indicated by their resistance to antibiotics (Figure 6C). These observations provide one of the more solid indications to the localization of live *F. tularensis* in cells of the infected host, and identify the RTDC as an *in vivo* niche for pathogen residence. The fact that most cells carry several intracellular bacteria probably reflects intracellular replication of LVS, rather than simultaneous uptake of several bacteria by an individual cell.

While MdLN DC appear to carry LVS, one cannot overlook the presence of a large extracellular bacterial load in the infected MdLN (Figure 6A). This finding underlines the long and unresolved debate on the interrelationship between the intracellular and the extracellular life styles of *F. tularensis*, and their relevance to pathogenesis. While extracellular bacterial trafficking *per se* cannot be excluded, one can envision an infection mechanism that involves uptake of LVS by DC in the airways [18],[21] and import of bacteria-harboring DC into the MdLN followed by apoptosis-mediated (our unpublished results and those of others [14]) release of bacteria from the cells. Such a model would imply an initial stage of intra-DC residence required to overcome early host defense mechanisms, which is then followed by an extracellular colonization process, and possibly re-infection of more cells

A major support for the function of RTDC as transporters of LVS comes from the in vivo viable staining experiments (Figure 7). Staining of infected airway cells with CMTMR allowed us to determine that a major fraction of the CD11b-sorted, LVS-carrying cells are newly-immigrating cells, recruited from the respiratory tract to the MdLN after infection (Figure 7). Moreover enumeration of intracellular bacteria revealed that the about 75% of the bacteria carried by CD11b-sorted cells actually reside in the newly-immigrated cells.

The preferential presence of intracellular LVS in newly-immigrating RTDC (Figure 7C) provides very strong support to DC-mediated, LVS trafficking. In order to address the less-likely possibility of preference in LVS uptake by the newly-immigrating within the MdLN, we have treated mice with inhibitors of DC migration. Trafficking of DC from the infection site is governed by a variety of mechanisms. The most characterized mechanisms relate to controlled change of the surface-displayed chemokine receptors repertoires. Other mechanisms involve sphingosine-1-phosphate [6],[54], scavenger receptor A [55], osteopontin [56] and prostaglandins [5],[42]. It should be noted however that these mechanisms do not act exclusively on DC migration, and often exhibit pleotropic effects. This led us to examine two independent experimental systems. One system is based on FTY720, which desensitizes the S1P receptor, and thereby inhibits lymphocyte migration [30]. The other system is based on BW254C, a prostaglandin D1 analogue which interacts with the cognate DP1 receptor to inhibition of DC migration [5],[42]. Choosing these two effectors allowed us to use a drug that hampers positive migration signals, as well as an agonist that activates a physiological migration-impairing signal.

In spite of the major difference in their mode of action, treatment with either FTY720 or BW245C at the early stages of infection resulted in similar effects, impairment of both RTDC recruitment and LVS colonization of the MdLN (Figure 8 and Figure 9). Interestingly, the effect of FTY720 treatment on RTDC migration-impairment was more pronounced than that of BW245C (Compare Figure 8A and 8B and Figure 9A). This was translated into a more effective inhibition of bacterial dissemination by FTY720 than by BW245C (Compare Figure 8D and Figure 9B), providing additional support to the linkage between RTDC and LVS trafficking.

Instillation of each one of the migration-impairing agents to airways of infected mice prolonged disease progression. We chose, however, to concentrate on BW254C which is a drug of short-residence, and not on FTY720 which has long term effects, and therefore could influence later stages of disease. Instillation of the BW254C on days 0 and 1 of infection delayed the onset of morbidity by two days, and delayed the time of death by one day (Figure 9C and 9D). This again argues for a DC-driven bacterial spreading.

Taken together, all the observations presented here suggest that *F. tularensis* can inhabit DC *in vivo*, and DC migration can play a role in enhancing the invasiveness of the pathogen. In addition, this study provides guidelines to the development of a novel potential therapeutic strategy against respiratory tularemia. A treatment, based on impairment of DC trafficking could delay the onset of disease and provide an adequate window for the identification and the application of a suitable antibiotic treatment.

## Materials and Methods

### Bacteria preparation

*Francisella tularensis* live vaccine strain (ATCC 29684) stocks were plated on GCHI agar (GC Medium base, Difco, supplemented with 1% hemoglobin and 1% Iso-Vitalex BD, France). Working stocks were prepared from single individual colonies exhibiting the large-light phenotype [57].

For cell and animal infection experiments, bacteria were grown at 37°C to mid log phase (optical density of 0.1–0.2 at 660 nm) in TSBC (TSB Difco, supplemented with 0.1% cysteine) in a gyrostatory shaker. Bacteria were washed and then re-suspended at the desired concentration in either PBS for animal infection experiments, or RPMI 1640 medium (see below), devoid of antibiotics, for cell infection experiments.

Killed bacterial suspension were generated by incubating growth cultures, overnight, at room temperature in the presence of 0.4% formaldehyde, followed by extensive washing with PBS.

### Eukaryotic cell cultivation

BMDC were generated essentially according to the method developed by Lutz et al. [58] as described in detail previously [34]. More than 95% of the cells were CD11c positive as assessed by flow cytometry, indicating effective differentiation into DC.

BMDC as well as the J774A.1 macrophage–like cells were grown in RPMI 1640 medium supplemented with 10% FCS, 2 mM L-glutamine, 1 mM sodium pyruvate, 1% v/v MEM-EAGLE non-essential amino acid solution, 100 U/ml penicillin, 100 µg/ml streptomycin and 50 µM β-mercaptoethanol; all these components were supplied by Biological Industries (Beit Haemek, Israel).

### Cell Infection

BMDC (10^6^ cells/well in 24 well plates in supplemented RPMI devoid of antibiotics) were infected by pulsing with bacteria at an MOI (multiplicity of infection) of 200. Infection was initiated by spinning (140 g, 5 min) bacteria onto plated cells (this is referred to as time point 0 of infection). Pulsed cells were incubated at 37°C, 5%CO_2_ for 1 h before adding gentamicin (Sigma) at a concentration of 2 µg/ml. Incubation was then continued for additional 23 hours prior to analysis. In an alternative protocol, gentamicin-containing medium was replaced by fresh gentamicin-free medium after 2 hrs. This had no effect on bacteria counting. It should be pointed out that extracellular LVS did not propagate in the eukaryotic-cell growth medium, as noted by others as well [13],[59].

### In vitro transmigration assay

Infected cells were resuspended in RPMI containing 1% FCS to a concentration of 10^7^ cells/ml and were placed (10^6^ cells/well) in the upper compartments of Transwell migration chambers (Costar 3421, Corning, NY). CCL19 (R&D Systems) diluted to concentrations of 200 ng/ml in RPMI+1% FCS was placed in the lower compartments to induce CCR7-dependent chemotaxis. Medium alone served to evaluate CCR7-independent migration. DC were allowed to migrate through a polycarbonate (5 µm pore size mesh) at 37°C for 2 h, and cells migrating to the lower compartment were counted under light microscope. The experiments were performed in triplicates and migration was determined by calculating the percentage of migrating cells relative to input. Lipopolysaccharide (LPS) pulsing was conducted by application of 1 µg/ml of *Escherichia coli* LPS (Sigma).

### Animal infection and isolation of cells

C57BL female mice (8–10 weeks old) were used in most infection experiments. Some experiments were repeated using BALB/c mice as indicated. Mice anesthetized with ketamine/xylazine were infected intranasally by careful application of 25 µl LVS suspension at the desired concentration.

Bronchoalveolar lavages were performed on anesthetized mice through a 23-gauge catheter inserted into the trachea. Doses of 1 ml cold PBS were infused into each mouse and then aspirated from the airways. Animals were sacrificed by cervical dislocation and the desired organs were collected. Isolated organs were minced and treated with Liberase Blendzyme 3 (Roche) at final concentration of 2 µg/ml for 30–60 minutes at 37°C, followed by five minute treatment with 100 U/ml of Dnase I (Boehringer Mannheim). This was followed by passage through a cell strainer to obtain single cell suspension.

All experiments reported here were conducted in compliance with the guidelines of the animal use committee at the Israel Institute for Biological Research and are in accordance with the Animal Welfare Act.

### FTY720 and BW245C administration

FTY720 and BW245C were both purchased from Cayman chemicals (Ann Arbor, MI). FTY720 was diluted to a concentration of 40 µg/ml in PBS containing 10% ethanol. Twenty-five µl of the FTY720 solution (final amount of 1 µg) were administered to anesthetized mice by intranasal instillation at day zero (15 min prior to bacterial infection)

BW245C was diluted to a concentration of 0.4 mM in 0.3% DMSO in water, immediately prior to use. Twenty-five µl of the agonist solution (final amount of 10 nmol) were administered to anesthetized mice by intranasal instillation on day zero and on day 1 post infection. Carriers alone were distillated into mock treated animals

### Enumeration of cell-associated bacteria

Infected cell suspensions were submitted to centrifugation (140 g, 10 min), followed by two washes with PBS, in order to remove non-associated bacteria. When indicated, cells were incubated at 37°C for 30 min in the presence of 20 µg/ml gentamicin, followed by centrifugation and washes for gentamicin removal. Cells were lysed with either 0.1% deoxycholate (DOC) for 2 minutes or alternatively with 0.1% saponin for 30 minutes at 37°C. Bacterial suspensions were submitted to intensive mixing prior to serial dilution and plating on GCHI agar.

### Flow cytometry

Washed DC were incubated with PE or APC conjugated antibodies against CD11c (Clone N418), CD11b (clone M1/70), CD40 (clone 1C10), CD83 (clone Mitchel-17) and CD86 (clone GL1), as well as with the appropriate isotype-matched control antibodies. Reagents were purchased from eBioscience (San Diego CA). Staining was performed using standard incubation protocols (30 min at 4°C) except for CCR7 staining which was conducted at 37°C as indicated by the manufacturer. In all staining protocols, FcR was blocked prior to staining with FCR Block Reagent (Miltenyi Biotech, Germany), according to the manufacturer's protocol. Cells were collected on a FACSCalibur cytometry (Becton & Dickinson), excluding events smaller than 200 on the FSC.

### Magnetic cell sorting

Target cells were separated from the lymph node single cell suspension by magnetic microbeads carrying either anti-CD11c or anti CD11b antibodies (Miltenyi Biotech,

Germany), using the manufacturer's instructions. Prior to separation, cell suspensions were treated with the FcR Block Reagent (see above). About 10^8^ cells (pool of 8–10 lymph nodes) were then incubated with 100 µl of the microbead suspension for 15 min on ice, and washed to remove excess of free beads. Cells were passed through a column attached to a magnet and washed to separate bound and unbound cells. Out of 10^8^ cells submitted to sorting, about 10^6^ cells were bound to either anti-CD11c or anti-CD11b microbeads

### Monitoring in vivo migration of airway cells

Migration of cells from the airways to the peripheral lymph node was evaluated by tracking cells labeled by viable staining [29],[34]. Briefly, the orange cell tracer CMTMR (Molecular Probes, OR) was diluted in RPMI to a concentration of 8 mM and 30 µl/mouse were administered intranasally to mice anesthetized with ketamine/xylazine. Five hours later mice were instilled with 5×10^6^ bacteria per mouse (25 µl of bacterial suspension in PBS). At the indicated time post addition of bacteria, MdLNs were isolated, shredded and treated with 2 µg/ml Collagenase-D (Roche) for 30 min at 37°C. Cells were then passed through a 70 µm nylon mesh to yield a single-cell suspension, and analyzed by FACS.

### In situ visualization of cell-associated bacteria

Tissues or cells infected by LVS were examined for the presence of bacteria by fluorescent staining. J774A.1 cells were cultivated and infected in chamber slides and fixed with 3.7% formaldehyde. DC suspensions derived from bone marrow or from lymph nodes were placed in LabTekII chambered glass slides which are capable of binding semi-adherent cells (Nunc, Roskilde, Denmark). Cells were incubated for 20 minute at 37°C to allow binding. The bound cells were fixed with 3.7% formaldehyde in PBS for 30 min, followed by washing with PBS.

Dissected MdLNs were infiltrated with OCT (Sakura, The Netherlands), snap frozen in liquid nitrogen and transferred to storage at −70°C. Eight-micrometer cryostatic sections were cut and mounted on SuperFrost Plus slides (Menzel-Galaser, Germany). Slides were then fixed by dipping in cold acetone (−20°C) for 1 min. Fixed slides were blocked with either 0.5% BSA in PBS in the case of infected cell preparations, or with Rodent Block M (Biocare Medical, CA), for infected tissue. Hyper-immune antiserum of rabbits immunized with formalin killed LVS diluted 1/300 served as primary antibody, while normal rabbit serum served as negative control. Texas-Red or FITC-conjugated goat anti rabbit antibodies (Molecular Probes, OR) served as second antibody. Stained specimen were examined with an Axiovert 200 inverted microscope (Zeiss) equipped with an AxioCAM MRc5 digital camera (Zeiss).
